# Information Reconstruction of Student Management Work Based on Association Rules Mining

**DOI:** 10.1155/2022/2318515

**Published:** 2022-04-06

**Authors:** Yong Xiang, Chun Shuai, Yin Li, Yutong Zhang

**Affiliations:** ^1^Chengdu Normal University, Sichuan 611130, China; ^2^Sichuan University, Sichuan 610065, China; ^3^Chengdu Normal University, Sichuan 611130, China; ^4^Sichuan Business Vocational College, Sichuan 611130, China

## Abstract

In recent years, as the country has paid more and more attention to the education, informatization of student management has become more and more important. This article aims to study how to reconstruct the informatization of student management which is based on association rule mining. This article mainly introduces association rule mining and student management informationization. Based on data mining, an algorithm for association rules is proposed, and the algorithm is used to mine student management informationization. From the data in the experiment, it can be seen that the efficiency of traditional student management is between 25% and 35%, whereas the efficiency of student management information based on association rules is between 64% and 72%. It can be seen that the efficiency of student management work combined with association rule mining is significantly higher than that of traditional management methods. From the data, we can see that in 2017, the development trend of colleges and universities adopting information management rose from about 5.4% to about 11%, and the development trend of colleges and universities adopting information management rose from about 7.5% to about 33% in 2018. In student management, the simplification of information can effectively improve the efficiency of student management, so the reconstruction of student management information based on association rule mining has become very important.

## 1. Introduction

In the case of managing student information, the previous database technology was limited to simple information operations such as query and deletion. In the traditional database technology, it is difficult for the school management to find the required information, and the efficiency of data usage is also very low. Based on this, association rule data mining technology is used to manage the information of school students, reducing the intensity and complexity of manual operations, ensuring the efficiency and quality of information management, and providing a better foundation for school management. Association rule mining is one of the research focuses and hotspots in the field of data mining technology, and it has a wide range of applications in various industries. Apriori algorithm is one of the representative algorithms of association rules, and its performance is directly related to the efficiency and conclusion of association analysis.

Today's information technology provides schools with modern office equipment, improves office efficiency, and makes student management more efficient and convenient. Therefore, student information management is a unified management of data, network, and standardization. Informatization of student work is an inevitable requirement for innovative college student work under the new background. Only by continuously promoting and deepening the informatization of student work can university student work meet the challenges of the new era.

The innovations of this article are as follows:

1. The theoretical knowledge of association rule mining and student management informationization is introduced, and the association rule mining algorithm is used to analyze how association rule mining can play a role in the research of student management information reconstruction.
2. It analyzes the traditional methods of student management and the informatization of student management based on association rule mining. Through experiments, it is found that the informatization of student management based on association rule mining is more conducive to the development of college student management.

## 2. Related Work

As the country pays more and more attention to education, the informatization of student management has also become very meaningful. Jacksi et al. found that work management plays an important role in every organization. It directly affects the work efficiency of educational institutions, the learning efficiency of students, and the management efficiency of other management organizations. Students must maximize the speed of their management work. He found that managing student attendance during lectures has become a daunting challenge. So he proposed an efficient Web-based attendance management system application designed to track and manage students' activities in the classroom. But the scholar did not give a specific description of the system, so it is impossible to confirm whether the system has this function [1]. Lakhno proposed an informatization object with intelligent support subsystems, so as to achieve the purpose of the protection and control system architecture, which is used to make decisions on the operation and management of network protection. He developed a network protection operation management model using informationized objects and formed a reasonable protection method and mechanism. But he did not verify the reliability and authenticity of the method through specific experiments [2]. Buczak and Guven found that there is a great correlation between network analysis machine learning and data mining methods used to support intrusion detection. But at the same time, he also discovered that network analysis machine learning and data mining methods that support intrusion detection are facing threats to network security. He gave some suggestions to solve the network threats faced by the two methods. But his point of view is too vague, he did not specifically describe the relationship between the two, as well as specific measures and suggestions to solve the challenges [3]. Sheu and Chu analyzed the influencing factors of consumer acceptance of social networking sites and applied data mining algorithms to calculate the correlation between these influencing factors and consumer acceptance to understand the relationship between them. He found that consumer acceptance has a lot to do with the enjoyment of sharing relevant information with others. However, he did not elaborate on the influencing factors of consumer acceptance of social networking sites, nor did he explain the relationship between consumer acceptance and their level of pleasure [4]. Czibula et al. proposed association rules as a new data mining concept, which can extend the traditional association rules to express common rules that persist between attributes in the data set. Czibula et al. proposed a further extension. His goal is to create a more expressive and stable method to detect relational association rules. He introduced an algorithm similar to Apriori, which can effectively discover the role of association rules in data mining. But he did not use specific experiments to verify the more stable method he created, so this conclusion is not very convincing [5]. Zou et al. discovered that the concept lattice has been used in the field of artificial intelligence knowledge discovery. He proposed a rule mining algorithm based on fuzzy algorithms. The experimental results show that data mining incorporating association rules is more efficient. His experiment did not have specific subjects, nor did he have specific experimental data to support [6]. Can and Alatas found that classic optimization algorithms are too inefficient in solving complex search and optimization problems. Therefore, they used the gravity search algorithm to explore the association rules in the numerical database. The algorithm can search for quantitative association rules from the database of the search space. In addition, the fitness function used in the algorithm is very flexible. In the process of rule mining, the range value of the attribute has been automatically adjusted, making the association rule very flexible. But he did not explain how to operate the search algorithm to make the association rules searched out [7]. Nasereddin discussed the process of using association rule model estimation and construction. He found that the scanning project does not need to rescan the original database after collecting the data, the association rules work more effectively in a conventional form, and it can save a lot of time compared with the previously used technology. Although his conclusion is not wrong, he did not describe the process of using association rule model estimation and construction, nor did he list the experimental data, which made the experiment not very reliable [8].

## 3. The Basic Concepts of Data Mining and Student Management Informatization

With the rapid development of information technology, the trend of campus informatization is gradually taking shape, and China has entered the era of standardized education management informatization construction to some extent [9]. Student management informatization plays an important role in the modernization of school management. It can effectively improve the efficiency of campus management. In the process of university informatization, a complete information management system is indispensable. The campus informatization is shown in Figure 1:

As shown in Figure 1, now, with the innovation of decision-making science and the continuous development of modern management theory, informatization has been gradually introduced into management work by most universities. These working methods have also changed from management methods based on past experience to scientific management methods based on modern management theories [10].

Using data mining technology to analyze the educational administration data of students and teachers, we can find useful rules among them. These laws can guide the management of the school [11]. Data mining is shown in Figure 2.

As shown in Figure 2, with the accumulation of data, the abolished data becomes less and less useful for actual work. In the spatial sense, the accumulation of data takes up more and more storage space [12]. In the application of traditional data analysis and processing methods, the collection of these data cannot be effectively processed. Now the university's management information system is still traditional, and the low reliability of this information is directly related to work efficiency. In order to effectively solve these problems, it is necessary to reconstruct the informatization of student management by mining based on association rules.

In recent years, modern information technology has continued to advance, and various technological applications based on big data have become market hotspots. By applying big data to product marketing, customer experience improvement, risk control, and other aspects, good results have been achieved. Therefore, data mining will be applied to more and more industries in the future. With the popularization of large-scale databases and the rapid expansion of the Internet, the amount of data stored in databases around the world is rapidly increasing, which also means that the work is becoming more and more intense and difficult. The emergence of the field of data mining can discover knowledge methods from these huge data [13]. The data mining process is shown in Figure 3:

As shown in Figure 3, data mining not only helps people extract the knowledge of interest from the database but also helps to analyze the data to various degrees. Therefore, the data in the data warehouse can be further analyzed, and it can also be used to further predict future management trends [14].

As long as social networks and mobile interactive networks are involved, the information management of the university must keep pace with the times. In order to realize the new exploration of the depth and breadth of college student management, scholars continue to explore new areas [15]. The informatization process of student management based on data mining is shown in Figure 4:

As shown in Figure 4, effectively manage students in accordance with the needs of society for talents, improve the security of student management and student information in the era of big data, so that the school can take more convenient and effective methods when accessing student-related information [16].

As the scale of data collected and stored in the database becomes larger and larger, people are paying more and more attention to digging out relevant knowledge from these data.

## 4. Dynamic Association Rules and Multiscale Association Rules Based on Data Mining

### 4.1. Dynamic Association Rules Based on Data Mining

Data mining is an important data analysis technology, and association rules is a descriptive data mining. The algorithm of association rules is an unsupervised learning method. Dynamic association rule mining is to further describe the characteristics of rules and data on the basis of ordinary association rules. A dynamic association rule is a type of association rule that can describe independent changes over time. The specific instructions are as follows: setting up the project set, collect task-related transaction data set *D* in the period *t*, and *n* is the time series [17]. The dynamic association rule structure is shown in Figure 5:

As shown in Figure 5, the rule in transaction set *D* has a support degree of *S*, *S* is the percentage of *X* ∪ *Y* in the total database *D*, which is the probability *P*_*D*_(*X* ∪ *Y*). That is, the sum of the percentages of *X* ∪ *Y* contained in each subdata set in the total data set *D*, the calculation formula of *S* is as follows:

(1) $$\begin{array}{c} s=\sum_{i=1}^{n}\left[P_{D}{\left(X\cup Y\right)}_{i}\right]. \end{array}$$

Among them, *P*_*D*_(*X* ∪ *Y*) represents the item set contained in data subset *D*_*i*_, and *X* ∪ *Y* represents the proportion of the number of transactions in the total number of transactions in data set *D*.

The rule in transaction set *D* has a confidence level of *C*, which is the transaction that contains *X* in *D* and also contains the percentage of *Y*. That is, the sum of the percentages of transactions containing *X* ∪ *Y* in each subdata set relative to transactions containing *A* in *D*, and the calculation formula for *C* is as formula:

(2) $$\begin{array}{c} C=\sum_{i=1}^{n}\left[P_{D}\left(Y_{i}|X\right)\right], \end{array}$$

where *P*_*D*_(*Y*_*i*_*|X*) represents the ratio of the number of transactions of item set *B* in data subset *D*_*i*_ to the number of transactions of item set *A* contained in the entire data set *D*.

*S*_*i*_ corresponds to the probability *P*_*D*_(*X* ∪ *Y*) mentioned in the definition of association rules, so there is formula:

(3) $$\begin{array}{c} S_{i}=\frac{f_{i}}{m},\;i\in \left\{1,2,\ldots ,n\right\}. \end{array}$$

The support degree of item set *X* ∪ *Y* is denoted as *S*, and then, there is formula:

(4) $$\begin{array}{c} S=\sum_{i=1}^{n}S_{i}. \end{array}$$

Setting the minimum support to min_sup, then when *s* ≥ min_sup, itemset *X* ∪ *Y* is the dynamic frequent itemset. Formula (4) given above uses the value of the support to represent the elements of the support vector, but in some cases, it is more appropriate to use the item set frequency to represent the support vector [18]. A support vector is expressed as following formula:

(5) $$\begin{array}{c} SV=\left[f_{1},f_{2},\ldots ,f_{n}\right]. \end{array}$$

Similarly, when *s* ≥ min_sup, itemset *X* ∪ *Y* is a dynamic frequent itemset.

The original definition of this calculation method does not reflect the support measure of item set *X* ∪ *Y* in each subdata set, but can only provide the ratio of the frequency of *X* ∪ *Y* in the subdata set to the total data set [19]. From the perspective of information theory, the information provided by SV and CV is the same, so the information of CV is redundant. In view of the above problems in dynamic association rules, SV and CV are redefined, as described in formula:

(6) $$\begin{array}{c} \text{SV}=\left[s{\left(X\cup Y\right)}_{1},s{\left(X\cup Y\right)}_{2},\ldots ,s{\left(X\cup Y\right)}_{n}\right]. \end{array}$$

The value of each element of the support vector and trust direction obtained according to the above definition is consistent with the previous definition of support and trust, which is very helpful for recording relevant information of association rules.

### 4.2. Multiscale Association Rule Algorithm Based on Data Mining

Scaling theory has been introduced into the field of data mining, but people's research on it is still not deep and complete enough, and it lacks universal theories and methods. With the deepening of big data processing applications, its research becomes more urgent. Aiming at the above problems, researches on universal multiscale data mining theories and methods are carried out. Multiscale data mining can accomplish the tasks of multiscale realization of data and multiscale realization of knowledge [20]. Multiscale data mining is shown in Figure 6:

As shown in Figure 6, in many cases, data can only be represented or divided by a single scale. Therefore, the association rule mining uses the frequent item sets in the data set of the descendant ratio, thereby deriving the frequent item sets in the data set of the ancestor ratio [21].

When mining the descendant-scale data set *ds*_*h*_ − *v*^2^ with the minimum support min_sup, use the calculated minimum support to mine each descendant-scale data set, as shown in the following formula:

(7) $$\begin{array}{c} \min\_\sup_{i}=\min\_\sup-\sqrt{\frac{1}{2\left|ds_{h}-v^{2}\right|}\cdot In\frac{1}{p}}. \end{array}$$

The Jaccard similarity coefficient is used to compare the similarity and difference between a limited sample set. The larger the Jaccard coefficient value, the higher the sample similarity. From a statistical point of view, frequent item sets are the statistical results of the data set, and to a certain extent, they represent the distribution and characteristics of the data set itself. Generally, the Jaccard similarity coefficient is applied to actual research in the field of data mining, as shown in the following formula:

(8) $$\begin{array}{c} \text{Jaccard}\left(X,Y\right)=\frac{\left|X\cap Y\right|}{\left|X\cup Y\right|}. \end{array}$$

Using formula (8) to calculate the (*X*, *Y*) Jaccard similarity coefficient and use this similarity coefficient as an estimate of the similarity between data sets *X*∩*Y*.

Using the weighted average method, the estimated value of the unknown support count supcnt_*i*_ in the candidate set is as follows:

(9) $$\begin{array}{c} \text{est}\_\sup{\text{cnt}}_{i}=\left|ds_{h}-v^{2}\right|\cdot \frac{1}{m}\sum_{j=\alpha }^{\beta }M_{ij}. \end{array}$$

The multiscale association rule mining algorithm mainly uses the reciprocal distance weighting method in the spatial interpolation method for reference. The reciprocal distance weighting method is often compared with the Kriging method. It can be estimated with data sets of different distance points in a certain range around, the farther the data set is from the estimated point, the less effective it is. The basic idea is first determine the influence weight of the neighboring sampling points to be interpolated and then use the relevant attribute values of the sampling points and the corresponding weights to calculate the estimated value of the attributes of the interpolated points [22].

Among them, *A*_*i*_(*i*=1,2,…, *n*) is a series of sampling points or observation points within the research range, *Z*(*A*_*i*_) is the observation value corresponding to *A*_*i*_, *λ*_*i*_ is the weight of *A*_*i*_ to be interpolated point *A*_0_, and the value of to be interpolated point *A*_0_ is as shown in the following formula:

(10) $$\begin{array}{c} Z\left(A_{0}\right)=\sum_{i=1}^{n}\lambda_{i}Z\left(A_{i}\right). \end{array}$$

Using the reciprocal distance weighting method to calculate the support of the candidate item set obtained from the upper-level data set in the target lower-level data set and filter the frequent item sets in the final lower-level data set to generate association rules, as shown in the following formula:

(11) $$\begin{array}{c} \lambda_{i}=\frac{d_{io}^{-\mu }}{\sum_{i=1}^{n}d_{io}^{-\mu }}. \end{array}$$

The calculation of weight *λ*_*i*_ in the reciprocal distance weighting method only considers the distance between the observation point *A*_*i*_ and the point to be interpolated *A*_0_. The greater the *μ*, the greater the weight of the observation point from the point to be interpolated.

Calculating the similarity between the upper-scale data sets, construct the sibling-scale data set similarity matrix Sim_Martrix, where *M*_*ij*_ represents the sibling-scale data set, as shown in the following formula:

(12) $$\begin{array}{c} M_{ij}=\text{Jaccard}\left[A,B\right]=\frac{\left|A^{i}\cap B^{i}\right|}{\left|A^{i}\cup B^{i}\right|}. \end{array}$$

The weighted average method uses several past observations of the same variable arranged in chronological order and takes the number of occurrences of the chronological variable as the weight to calculate the weighted arithmetic average of the observations, use this number as a trend forecasting method to predict the predicted value of the variable in the future. Using the weighted average method, calculate the unknown support est_sup_*i*_ estimated value in Sim_Martrix corresponding to the candidate item set, as in the following formula:

(13) $$\begin{array}{c} \text{est}\_\sup_{i}=\frac{1}{m}\cdot \sum_{j=1}^{m_{x}}M_{ij}\cdot \sup_{j}. \end{array}$$

From the perspective of algorithm analysis, the realization of multiscale association rule mining algorithms to data sets with multiscale characteristics is more practical in terms of processing and results, especially when the informatization of management work is required.

The degree of support refers to the number of transactions of a specific item set *A* in the transaction database *D*, denoted as *δA*, so that the support rate Support(*A*) can be calculated, as in the following formula:

(14) $$\begin{array}{c} \text{Support}\left(A\right)=\frac{\delta A}{\left|D\right|*100\%}. \end{array}$$

Confidence degree refers to the percentage of things in *D* that include *A* under the premise that they also include *B*. This condition is referred to as *P*(*b|a*), which is recorded as: confidence(*a*⟶*b*), as in the following formula:

(15) $$\begin{array}{c} \text{confidence}\left(a⟶b\right)=\frac{\text{support}\left(a\cup b\right)}{\text{support}\left(a\right)*100\%}. \end{array}$$

In statistics, the confidence interval of a probability sample is an interval estimate of a certain set of parameters of the sample. The minimum confidence level is an important parameter for generating association rules, and support and confidence are two important concepts that differ in association rule mining. The main function of the former is to measure the importance of transaction data based on statistical principles, while the latter is to measure the credibility of the rules.

Dividing the data into *n* blocks, and the sum of the local minimum support in *n* nodes is the global minimum support, so the local minimum support is the product of the global minimum support and the number of transactions in the node data block, expressed as min_sup, as in the following formula.

(16) $$\begin{array}{c} L\min\_\sup=\min\_\sup^{*}\frac{\left|\text{BR}\right|}{n}. \end{array}$$

Both the local average weight and the global average weight represent the degree of relevance of a certain item combination within the item set, so the quotient of the local average weight and the local support count is expressed by *B*.LaverageWeight, as in the following formula:

(17) $$\begin{array}{c} B.\text{LaverageWeight}=\sum A_{i}\frac{\text{Weight}}{A}, \end{array}$$

where Weight is the local support count of *B*, 1 ≤ *i* ≤ *A*.

When merging the frequent item sets calculated on each node, the frequent item sets on all nodes are regarded as part of the global frequent item sets, and the frequent item sets only on some nodes are regarded as the global candidate frequent item sets.

First scan the original database *D*, traverse all the item sets in the transaction, and count their support, that is, the number of occurrences. The support count of record item set A is expressed as *A*.sup, as in the following formula:

(18) $$\begin{array}{c} A.\sup=\text{sum}A\left(T_{i}\right). \end{array}$$

In formula (18), *i*=1,2,…, *n*; *n* is the number of transactions in the data, and sum*A*(*T*_*i*_) is the sum of the number of occurrences of item sets in all transactions.

Calculating the support count and average weight of each candidate item set. The global average weight is the quotient of the weights of all items in item set *A* and the global support count, represented by *A*.GaverageWeight, as in the following formula:

(19) $$\begin{array}{c} A.\text{GaverageWeight}=\sum \min\frac{\left(A_{i}\text{Weight}\right)}{A.G\sup}. \end{array}$$

Among them, *A*.*G*sup is the global support count of itemset *A*. All item sets satisfying the minimum average weight and minimum support at the same time are another part of the global frequent item sets, and these two frequent item sets are all the global frequent item sets.

## 5. Experiment and Analysis of Student Management Informatization

### 5.1. Traditional Student Management Work and Student Management Work Based on Association Rules

The advantages of student information management are that information can circulate quickly, get accurate information, improve work efficiency, facilitate communication, and obtain information and grasp the basic status of students at any time, and the management is convenient and simple.

Colleges and universities are also undergoing rapid changes. The enrollment scale continues to expand, the number of students at school has doubled, the campus is rapidly expanding, and the development of multidisciplinary cross-disciplinary development. These changes have brought certain challenges to the management of college students. Facing these difficulties and challenges, how to solve the above problems has attracted more and more colleges and colleagues' attention. Colleges and universities must adapt to these changes and come up with more efficient solutions. At present, most colleges and universities tend to gradually solve the above problems through the construction of informatization.

This article compares the development trend of informatization management adopted by colleges and universities in 2017 and 2018, as shown in Figure 7:

As shown in Figure 7, with the popularization and development of the Internet, the work patterns of all walks of life have changed, and the work efficiency of all walks of life has been improved, and it has gradually penetrated into the student management work of the university. If the information mode is used, the management of students will be more efficient, and the pressure on employees will be reduced, forming a more scientific student management system.

This article compares the traditional informatization efficiency of student management with that of student management based on association rules, as shown in Figure 8.

As shown in Figure 8, effective use of data accumulated by universities to mine potential knowledge to help managers make constructive decisions is very important in the field of education. It can be seen from Figure 8 that the standardization of traditional student management information is between 25% and 32%, and the standardization of student management information based on association rules is between 65% and 68%. The university has accumulated a large amount of data in education and management business for many years. It can not only effectively improve the educational efficiency of teachers but also provide a scientific basis for educational administration and teachers' educational methods through inspection and feedback information, which will improve the standardization, service, and scientific nature of university management.

### 5.2. The Efficiency of the Association Rules before and after the Improvement in the Informatization of Student Management

So it takes a lot of time to mine candidate item sets and repeatedly scan huge databases.

This article compares the operation of the association rule algorithm before and after the improvement in different data sets, as shown in Tables 1 and 2.

From the data in Tables 1 and 2, it can be seen that the working efficiency of the improved association rule algorithm under different data sets is between 34% and 37%, the working time is between 12.4 seconds and 14.5 seconds, and the number of rules is between 5.6 and 6.8. The working efficiency of the improved association rule algorithm under different data sets is between 35% and 39%, the working time is between 11.7 seconds and 13.6 seconds, and the number of rules is between 6.2 and 6.5. It can be known that the efficiency of the improved association rules is about 1% higher than the efficiency of the association rules before the improvement, so different data sets have little effect on the improved association rules.

In order to verify the reliability of the experiments, this article compares the operation of the improved association rule algorithm under different support thresholds before and after the improvement, as shown in Tables 3 and 4.

According to the data in Tables 3 and 4, the working efficiency of the improved association rule algorithm under different support thresholds is between 29% and 39%. The working time is between 11.7 seconds and 12.9 seconds, and the number of rules is between 6.2 and 7.6. The working efficiency of the improved association rule algorithm under different data sets is between 48% and 69%, the working time is between 8.5 seconds and 12.3 seconds, and the number of rules is between 6.2 and 7.3. It can be known that the efficiency of the improved association rules is about 19% higher than the efficiency of the association rules before the improvement, so different support thresholds have a great impact on the improved association rules.

This article compares the execution time and work efficiency of the association rule algorithm before and after the improvement, as shown in Figure 9.

It can be seen from Figure 9 that under the same amount of data and different degrees of support, through the comparison of the length of execution time and the efficiency of the algorithm before and after the improvement, it is known that the execution time of the association rule algorithm before the improvement increased from 32 seconds to 37 seconds, and the execution time of the improved association rule algorithm dropped from 19 seconds to 17 seconds. As the amount of data increases, the working efficiency of the association rule algorithm before the improvement is not obvious or even has a downward trend. However, the working efficiency of the improved association rule algorithm increases significantly with the increase in the amount of data.

The informatization of management work has had a great impact on student management, and its impact is mainly as follows:

1. An effective platform is constructed, communication is strengthened, and communication is promoted. The most effective way to properly implement management at a university is to communicate, so that communication channels and mechanisms that can correctly convey the opinions of students and employees can be established.
2. Saving time and cut costs. If use the information model, it can effectively reduce the work steps. In the previous method, it was necessary to communicate face to face, which required adjustment of the time and place of the two. Also, information-based management can effectively reduce intermediate links, directly use the network operating system to collect opinions, and organize them in the shortest time, which can solve problems in a timely manner. This not only saves time effectively but also saves costs in various aspects.

## 6. Discussion

This article analyzes how to reconstruct the informatization of student management based on association rule mining. It expounds the related concepts of association rule mining and student management informatization, studies the related theories of data mining, and explores the method of reconstructing student management informatization. Also, through investigation method to discuss the importance of student management informatization and finally take the integration of association rules into student management informatization as an example to explore the relevance between the two.

This article also makes reasonable use of association rule mining algorithms. As the application range of association rule mining algorithms has become more extensive, and its importance has gradually become more prominent; many scholars have begun to match the theory of association rule mining algorithms with real-life application scenarios and put forward feasible algorithms. Association rule mining algorithm is a kind of mathematical operation. According to the calculation, it is indispensable for the research on the information reconstruction of student management work based on the association rule mining algorithm.

Through experimental analysis, this article shows that in today's rapidly developing social background, efficient student management has become more and more important, and the reconstruction of student management information based on improved association rule mining is of great significance.

## 7. Conclusions

This article mainly focuses on association rule mining and student management informatization. It extends from association rules to data mining and gives a detailed introduction to the theoretical knowledge of data mining and its role in student management. In the method part, this article studies dynamic association rules and multiscale association rule mining algorithms and uses this algorithm to conduct experiments. In the experiment part, the development trend of informatization of student management work in recent years was investigated. The survey results found that the development trend of informatization of student management has gradually increased in recent years, indicating that the informatization of student management has a great impact on colleges and universities. The traditional way of student management is not only inefficient but also wastes a lot of time. The informatization of student management work combined with association rule mining has become simpler, and the efficiency of student management work has also been improved. It can be seen that based on association, mining plays a huge role in the reconstruction of student management information.

## Figures and Tables

**Figure 1:** Application diagram of campus informatization.

**Figure 2:** Data mining structure diagram.

**Figure 3:** Data mining process.

**Figure 4:** Informatization process of student management.

**Figure 5:** Dynamic association rule structure.

**Figure 6:** Multiscale data mining.

**Figure 7:** The development trend of colleges and universities adopting informatization management from 2017 to 2018. (a) The development trend of colleges and universities adopting information management in 2017. (b) The development trend of information management in colleges and universities in 2018.

**Figure 8:** Comparison of the efficiency of student management in the two methods. (a) Traditional student management information efficiency. (b) Information efficiency of student management based on association rules.

**Figure 9:** Comparison diagram of association rule algorithms before and after improvement. (a) Association rule algorithm before improvement. (b) Improved association rule algorithm.

**Table 1:** The operation of the association rule algorithm before the improvement under different data sets.

Algorithm	Data set size	Mining efficiency	Operation hours	Number of rules
Before improvement	100	35	12.4	5.6
	200	37	14.5	5.9
	300	36	13.5	6.7
	400	34	13.9	6.8
	500	37	12.8	6.3

**Table 2:** The operation of the improved association rule algorithm under different data sets.

Algorithm	Data set size	Mining efficiency	Operation hours	Number of rules
After improvement	100	37	11.7	6.3
	200	39	13.6	6.2
	300	38	12.8	6.4
	400	35	12.4	6.3
	500	36	12.6	6.5

**Table 3:** The operation of the association rule algorithm before the improvement under different support thresholds.

Algorithm	Support threshold (%)	Mining efficiency	Operation hours	Number of rules
Before improvement	5	36	11.7	7.6
	10	29	12.8	7.4
	15	38	12.6	6.9
	20	39	12.9	6.3
	25	36	11.9	6.2

**Table 4:** The operation of the improved association rule algorithm under different support thresholds.

Algorithm	Support threshold (%)	Mining efficiency	Operation hours	Number of rules
After improvement	5	48	11.9	7.3
	10	52	12.3	7.2
	15	59	9.7	6.3
	20	65	9.3	6.6
	25	69	8.5	6.2

## Data Availability

The data sets used and/or analyzed during the current study are available from the corresponding author on reasonable request.
